# Meta-analysis of the effect of percutaneous coronary intervention on chronic total coronary occlusions

**DOI:** 10.1186/1749-8090-9-41

**Published:** 2014-02-28

**Authors:** Ruogu Li, Shuansuo Yang, Lei Tang, Yiqing Yang, Hui Chen, Shaofeng Guan, Wenzheng Han, Hua Liu, Jinjie Dai, Qian Gan, Weiyi Fang, Xinkai Qu

**Affiliations:** 1 Department of Cardiology, Shanghai Chest Hospital Affiliated to Shanghai Jiaotong University, NO.241, Huaihai Xi Road, Xuhui District, Shanghai 200030, China; 2 Department of Cardiology, Central Hospital, Fengxian District, Shanghai 201400, China; 3 School of Medical Graduate, Shanghai Jiaotong University, Shanghai 200025, China; 4 Department of Cardiovascular Research, Shanghai Chest Hospital Affiliated to Shanghai Jiaotong University, Shanghai 200030, China

**Keywords:** Coronary artery chronic total occlusion, Percutaneous coronary intervention, Meta-analysis

## Abstract

**Background and purpose:**

Coronary chronic total occlusion (CTO) is the last stage of coronary artery atherosclerosis. Percutaneous coronary intervention (PCI) is a therapeutic procedure used to recanalize vessels with total occlusion. However, successful recanalization of CTO is still not optimal, and the key influence factors are still uncertainty. Therefore, a scientific evaluation on the effective of PCI for CTO treatment is necessary.

**Methods:**

Relevant studies of PCI treatment for CTO were examined. Data were extracted and assessed by two independent clinical experts. Embase, PubMed and Medline et al. were used as database. The main research key words include “CTO”, “PCI”, “Stent”, “Reopen”, “long-term”, “follow-up” and “outcome”. Quality assessment was carried out according to the Cochrane Handbook. The selected data were pooled and analyzed using fixed-effect model and random-effect model. Heterogeneity was assessed using the *I*^2^ test, Q test, L’abbe and Galbraith. Comprehensive Meta -Analysis 2.0 and Metanalysis 1.0 were used for statistics analysis in this research.

**Results:**

A total of 16 articles involving 6695 cases in successful CTO recanalization (CTO success group) and 2370 cases in failed CTO recanalization(CTO failure group) were included in this research. Low CTO success was associated with elder age, previous coronary artery bypass graft surgery (CABG) history, multi-vessel diseases and right coronary artery disease lesion. Six follow-up variables including major adverse cardiac events (MACE), recurrent myocardial infarction (MI), all-cause death, incidence of angina, subsequent CABG and cumulative survival rate were found significantly reduced associated with CTO success.

**Conclusions:**

Clinical baseline characteristics such as age, previous CABG history and lesion baseline characteristics such as lesion length, multi-vessel diseases might be important factors influencing the successful rate of CTO recanalization. Compared to CTO failure patients, all six follow-up variables showed advantage for CTO success patients.

## Background

Coronary chronic total occlusion (CTO) is the last stage of coronary artery atherosclerosis, accounting for one third of the disease confirmed by coronary angiography [1]. CTO exists in about 50% of patients with coronary artery disease, which is often accompanied by complex lesions, in about 15% patients as reported, revealed by coronary angiography [2]. This disease can result in myocardium ischemia, myocardiolysis, reduction of the number of myocardial cells, ventricular remodeling which lead to decreased myocardium contractile, reduction of quality of life and poor prognosis [3]. Medication alone for CTO treatment does reduce the clinical symptom, but it has little effect on the long-term heart function and the improvement of the patients’ survival rate. Percutaneous coronary intervention (PCI) is a therapeutic procedure not only used to recanalize vessels with total occlusion [4], but also widely used in other aspects such as increase blood flow reperfusion, improve myocardial contractile and pump function [5], inhibit left ventricular remodeling and decrease adverse cardiac events [6]. However, PCI is considered not suitable for CTO lesions because of the lack in strong backup support by the guiding catheters or the difficulty in taking the contralateral coronary angiograms [7]. The success rate of CTO patients by PCI procedure is lower than that in non-CTO patients [8]. Revascularization for CTO lesions [9] is more difficult and influenced by baseline clinical characteristics, lesions level, intervention equipments and the manipulation techniques [10]. With the development of interventional technologies and physician’s manipulation techniques, the successful rate of PCI procedure on CTO lesions is significantly increased [8]. However, CTO recanalization is still accepted as an extremely challenging procedure in cardiovascular PCI treatments.

The success of the recanalization for CTO in coronary interventions is vital [11]. However, the long-term outcomes such as cumulative survival rate, major adverse cardiac events (MACE), incidence of restenosis and reocclusion are still under debate based on different procedures and techniques [12]. Therefore, it is critical to scientifically evaluate the effectiveness and influential factors for CTO interventional treatment.

In this study, publications on PCI procedure in CTO patients were systematically reviewed [13] and suggested potential influential factors that influenced successful rate and outcomes for PCI procedure [14].

## Methods

### Selection criteria for articles

Two investigators independently searched Embase, PubMed, Medline, Ovid, CCTR, CNKI, CMBdisc, and with additional manual search for related meeting abstracts and websites including American Heart Association American College of Cardiology, European Society of Cardiology, and national postgraduate thesis pool (from January 1990 to December 2009). The main research key words include “CTO”, “PCI”, “Stent”, “Reopen”, “long-term”, “follow-up” and “outcome”. No language restrictions were used. The inclusion criteria for selected studies comprised: 1) patients with CTO diseases, 2) comparisons of recanalization after PCI and unsuccessful recanalization and 3) the follow-up period of articles were at least one year. Studies with incomplete data or cases number less than 50 were excluded from the analysis.

### Data extraction

Clinical results with prespecified data forms were selected by two independent investigators. Meta-analysis was conducted by two independent clinical experts and the data was pooled by fixed-effect model and random-effect model [15].

### Quality assessment

Two independent investigators assessed the quality of eligible articles according to the Cochrane Handbook [16] with established methods. It includes 5 items: (i) Sequence generation; (ii) Allocation sequence concealment; (iii) Blinding of participants, personnel and outcome assessors; (iv) Incomplete outcome data; (v) Selective outcome reporting.

### Statistics analysis

The 95% confidence interval (CI) were calculated from abstracted dichotomous data of each study and pooled according to fixed-effects (inverse-variance weighted) and random-effects (DerSimonian and Laird) models. Statistical heterogeneity was assessed with Cochran’s Q via a chi-square test and quantified with the I^2^ test, P < 0.10 and I^2^ > 50% suggesting significant heterogeneity, I^2^ ≤ 25% considering low heterogeneity. Searching Software for analysis were Comprehensive Meta-Analysis 2.0 and Metanalysis 1.0.

## Results

A total of 16 reports [17-32] during 1990 and 2009 (randomized controlled trials and retrospective studies etc.) were included in consistency with the selection criteria. Totally 6695 cases in successful CTO recanalization (CTO success group) and 2370 cases in failed CTO recanalization (CTO failure group) were included in this study.

### Influential factors for CTO recanalization

In order to compare clinical and lesion baseline characteristics between CTO success group and CTO failure group, meta-analysis was performed on the studies of CTO revasculization with mean successful rate of 73.9% for CTO recanalization. Eight clinical baseline characteristics (including age, gender, hypertension, hyperlipidemia, diabetes mellitus, smoker, previous myocardial infarction history, previous coronary artery bypass graft surgery (CABG) history) and six lesion baseline characteristics (lesion length, left ventricular ejection fraction, multi-vessel coronary disease, left anterior descending artery lesion, circumflex artery lesion, right coronary artery disease lesion) were analyzed to assess discrepancies between two treatment groups. Among these, weighted average age difference between two groups was 0.083 (95% CI, 0.132 ~ 0.034, P = 0.001, heterogeneity, Q = 31.571, P = 0.005, *I*^2^ = 50.655%) (Figure 1), weighted average lesion length difference was -0.782 (95% CI, -1.499 to -0.065, P = 0.033, Q = 39.806 P < 0.001, *I*^2^ = 94.976%, Figure 2). The low CTO success rate was associated with previous CABG history (OR 0.707, 95% CI, 0.578 to 0.865, P = 0.001, Q = 1.962 P = 0.854, *I*^2^ = 0.00%, Figure 3) and multi-vessel diseases (OR, 0.649, 95% CI, 0.554 to 0.761, P < 0.001, Q = 26.943 P = 0.029, *I*^2^ = 44.326%, Figure 4). The other factors including gender, hypertension, hyperlipidemia, diabetes mellitus, smoker, previous myocardial infarction history, left ventricular ejection fraction, left anterior descending artery lesion and circumflex artery lesion did not affect the recanalization rate of PCI on CTO (P > 0.05).

**Figure 1:** Pooled results of the weighted mean difference of age of patients in CTO success groups and CTO failure groups.

**Figure 2:** Pooled results of the weighted mean difference of lesion length of patients in CTO success groups and CTO failure groups.

**Figure 3:** Pooled results of the effect of the history of CABG on patients in CTO success groups and CTO failure groups.

**Figure 4:** Pooled results of the effect of multi-vessel diseases on patients in CTO success groups and CTO failure groups.

### The long term effect of PCI on CTO recanalization

A total of 16 articles were studied on long term outcomes (follow up for more than one year) between CTO success group and CTO failure group. Six follow up variables including MACE, MI, all-cause death, angina pectoris, subsequent CABG and accumulative survival rate were analyzed. CTO success rate was associated with significant reduction in MACE (OR, 0.689, 95% CI, 0.488 to 0.971, P = 0.034, Q = 41.951 P < 0.001, *I*^2^ = 76.163%, Figure 5), MI (OR, 0.578, 95% CI, 0.387 to 0.864, P = 0.008, Q = 11.80 P = 0.107, *I*^2^ = 40.580%, Figure 6), all-cause death (OR, 0.501, 95% CI, 0.384 to 0.654, P < 0.001, Q = 28.283 P = 0.012, *I*^2^ = 51.02%, Figure 7), incidence of angina (OR, 0.477, 95%CI, 0.340 to 0.670, P < 0.001, Q = 12.977 P = 0.043, *I*^2^ = 53 .764%, Figure 8), subsequent CABG (OR, 0.212, 95% CI, 0.175 to 0.257,P < 0.001, Q = 9.873 P = 0.452, *I*^2^ = 0.00%, Figure 9) and cumulative survival rate (hazard ratio (HR), 0.595, 95% CI, 0.488 to 0.791, P < 0.001, Q = 11.714 P = 0.039, *I*^2^ = 57.317%, Figure 10).

**Figure 5:** Pooled results of major adverse cardiac events of patients in CTO success groups and CTO failure groups.

**Figure 6:** Pooled results of recurrent myocardial infarction of patients in CTO success groups and CTO failure groups.

**Figure 7:** Pooled results of all-cause death of patients in CTO success groups and CTO failure groups.

**Figure 8:** Pooled results of recurrent angina of patients in CTO success groups and CTO failure groups.

**Figure 9:** Pooled results of subsequent CABG of patients in CTO success groups and CTO failure groups.

**Figure 10:** Pooled results of long-term survival rate of patients in CTO success groups and CTO failure groups.

## Discussion

In this study, a scientific evaluation on the effective of PCI for CTO treatment was carried out. A total of 16 articles involving 6695 cases in successful CTO recanalization (CTO success group) and 2370 cases in failed CTO recanalization (CTO failure group) were included in this research. All the articles were used to identify the factors that influenced the PCI procedure outcome leading to a successful CTO recanalization or failed CTO recanalization. Finally, the clinical baseline characteristics such as age, previous CABG history and lesion baseline characteristics such as lesion length, multi-vessel diseases were considered being the important factors influencing the successful rate of CTO recanalization. Compared to CTO failure patients, the six follow-up variables (MACE, recurrent myocardial infarction, all-cause death, recurrent angina pectoris, subsequent CABG and accumulated survival rate) showed advantage for CTO success patients.

A lot of strategies and devices have been developed for a cure of CTO, but the success rate for each treatment is not consistent [33]. Previous study reveals that PCI significantly improved both the local and global function of the left ventricle in CTO patients [34]. Such procedure is beneficial for the symptom in selected patients [35]. However, NCDR (National Cardiovascular Data Registry) suggested that the attempt rate of PCI on CTO have not changed between 2004 and 2009 in the U.S., even though there are significant advance in the techniques in this area [36], indicating that risks under such procedure and factors affecting the success rate existed. Although the use of PCI for CTO increases recently [37], little systematic study directly compared the failed and success surgery cases with successful recanalization to identify the important factors under PCI. In this study, eight clinical baseline characteristics (age, gender, hypertension, hyperlipidemia, diabetes mellitus, smoker, previous myocardial infarction history and CABG history) and the and six lesion baseline characteristics (lesion length, left ventricular ejection fraction, multi-vessel coronary disease, left anterior descending artery lesion, Circumflex artery lesion and right coronary artery disease lesion) were revealed by directly compared the failed and success surgery cases with successful recanalization. The factors such as age, previous CABG history, lesion length and multi-vessel diseases might be important for the successful rate of CTO recanalization. Long-term patency after recanalization of CTO in patients with angina pectoris is associated with improvement in global and regional left ventricular function [38]. BEPM Claessen et al., [39] revealed that the presence of a CTO is associated with long-term mortality. In this study, six follow up variables including MACE, MI, all-cause death, angina pectoris, subsequent CABG and accumulative survival rate were analyzed by meta-analysis. CTO success was found to be associated with significant benefit in all these factors (Table 1), which were consistent with previous studies.

**Table 1:** Characteristics of 16 included studies

**Study**	**Year of publication**	**No. of patients**	**No. of patients with successful recanalization**	**Country**	**Occlusion time (month)**	**Clinical follow- up (year)**
Finci [23]	1990	200	100	Switzerland	3	2
Warren [18]	1990	44	26	Australia	1	2.6
Ivanhoe [19]	1992	480	317	America	3	4
Noguchi [20]	2000	226	134	Japan	3	4.3
Suero [21]	2001	2005	1491	America	1	10
Olivari [22]	2003	376	289	Italy	1	1
Hoye [8]	2005	871	567	Netherland	1	4.5
Drozd [24]	2006	459	298	Poland	1	2.5
Prasad [25]	2007	1262	914	America	3	10
Aziz [26]	2007	543	377	U.K.	3	1.7
Valenti [27]	2008	486	344	Italy	3	1
de Labriolle [28]	2008	172	127	America	3	2
Zhuyanbin [29]	2008	115	81	China	3	3
Chenshaoliang [30]	2009	152	132	China	3	1/3
Yixianhua [31]	2008	1604	157	China	3	3
Liubingwei [32]	2008	41	22	China	3	2

Although intervention studies that contain only randomized trials as observational studies are not designed for causal inference, observational studies itself also provide information that may suggest important message in certain circumstance [40]. Compared to the patients in CTO success group in our study, patients in CTO failure group were aged with severe lesion length and multi-vessel diseases. These negative effects made their cases more complicated and leaded to complications as well as the end of procedure ahead of time. These factors might be confounding variables for the analysis of the long term effects after PCI procedure. However, the result of clinical baseline characteristics such as age, previous CABG history, lesion length and multi-vessel diseases were not specific. There was no conclusion on how long of lesion length could be benefit for CTO recanalization, or how old of the patients will have higher successful rate of CTO recanalization. Moreover, limitations also existed in this study such as no bias test and text discrepancy. Meanwhile, a subgroup analysis of time effect on the involved studies was necessary.

## Conclusions

The factors including age and CABG history as well as the baseline lesion level (lesion length and multi-vessel diseases) might be the important factors influencing the successful rate of CTO recanalization. The in-hospital mortality, MACE, and incidence of subsequent CABG for PCI procedure were significantly lower in the CTO success group compared with those in the CTO failure group. All six follow up variables (MACE, recurrent myocardial infarction, all-cause death, recurrent angina pectoris, subsequent CABG and accumulated survival rate) showed an advantage for CTO patients with a successful recanalization of occlusions.

## Abbreviations

CTO: Coronary chronic total occlusion; PCI: Percutaneous coronary intervention; CABG: Coronary artery bypass graft surgery; MACE: Major adverse cardiac events; MI: Myocardial infarction; NCDR: National Cardiovascular Data Registry; PCI: Percutaneous coronary intervention; CI: Confidence interval.

## Competing interests

The authors declare that they have no competing interests.

## Authors’ contributions

RL, SY, LT carried out the studies, RL, HC, SG participated and drafted the manuscript. RL, WH, HL carried out the immunoassays. JD, QG, WF participated in the sequence alignment. RL, SG, HL participated in the design of the study and performed the statistical analysis. LT, SY, YY, WF conceived of the study, and participated in its design and coordination and helped to draft the manuscript. All authors read and approved the final manuscript.
